# Research on the Expression Level of Matrin-Type Zinc Finger Protein 4 Gene in T Cells of Thyroid Carcinoma Tissue

This article has been retracted.

**DOI:** 10.1155/2022/9884155

**Published:** 2022-08-18

**Authors:** Qian Zhang, Yingchun Song, Shengguang Chen, Zhongwei Lv

**Affiliations:** ^1^Department of Nuclear Medicine, Shanghai Tenth People, s Hospital, Tongji University School of Medicine, Shanghai 200072, China; ^2^Department of Endocrinology and Metabolism, Gongli Hospital of Shanghai Pudong New Area, Shanghai 200072, China

## Abstract

In order to analyze the expression level of zinc finger matrin-type protein 4 (ZMAT4) gene in T cells of thyroid carcinoma (TC) tissue and its clinical significance to prognosis of patients based on bioinformatics and reverse transcription polymerase chain reaction (RT-PCR), 389 TC patients with ZMAT4 gene and its corresponding survival and prognosis are searched by the Cancer Genome Atlas database. The expression of ZMAT4 gene is compared between normal thyroid tissue and TC tissue by RT-PCR. The relationship between ZMAT4 expression levels and clinicopathological parameters and baseline data is analyzed. The experimental results show that the low expression of ZMAT4 gene has an important relationship with the development of thyroid cancer, and real-time monitoring of ZMAT4 gene in TC patients can effectively evaluate the prognosis of patients.

## 1. Introduction

Thyroid cancer (TC), as the most common malignant tumor occurring in thyroid tissue, is mainly characterized by a hard and fixed mass in the thyroid gland accompanied by respiratory and swallowing difficulties [1]. At present, there are various theories about the pathogenesis of TC in clinical practice. Iodine deficiency, as one of the important factors leading to thyroid cancer, can stimulate hyperplasia and hypertrophy of thyroid follicle by reducing thyroxine synthesis. However, some scholars said that high iodine diet can also cause thyroid cancer. In addition, some scholars have proposed that radiation, sex hormones, and genetic factors are also the main causes of thyroid cancer [2, 3]. As a member of zinc finger (ZNF) family, zinc finger matrin-type protein 4 (ZMAT) plays an important role in eukaryotic cell proliferation, metastasis, and apoptosis as a transcription inhibitor. Among them, ZMAT4 is involved in the development of oropharyngeal squamous cell carcinoma and plays a role in the development of various tumor diseases due to its gene specificity [4]. This study uses bioinformatics methods to search ZMTA4 gene in T cells of TC patients from the Cancer Genome Atlas (TCGA) database. Reverse transcription polymerase chain reaction (RT-PCR) is used to detect the expression of this gene and analyze its clinicopathological characteristics and survival prognosis of patients with different TC, providing theoretical basis for the application value of ZMTA4 in the development and prognosis of TC.

The rest of this paper is organized as follows.  Section 2 discusses related work.  Section 3 analyzes the specific methods to obtain ZMAT4 data, and the relevant experimental indicators that should be observed in this study.  Section 4 shows the experimental results, and Section 5 concludes the paper with summary and future research directions.

## 2. Related Work

TC [5] as one of the most common malignant tumors in the endocrine system in clinical practice has a very high incidence worldwide. According to data, thyroid cancer patients are mainly young and middle-aged people, with the highest incidence in women, seriously threatening the life and health of patients [6, 7]. At present, clinical studies on thyroid cancer showed that the disease is characterized by rapid growth, easy metastasis, and strong recurrence, and its pathogenesis is not completely clear. Therefore, it is of great significance to further study the pathogenesis and predictive indicators of thyroid cancer and discuss new treatment plans for thyroid cancer [8]. As a member of the ZNF family, ZMAT4 gene has been localized in human 8p11.21. They contain 11 exons [9]. Related literature also showed that malignant tumors in the blood system are affected by copy number variation of ZMAT4. ZMAT4 copy number variation, independently or in combination with other markers, has certain positive significance as an indicator for the diagnosis of hematological malignancies [10]. Based on this, it can be speculated that ZMAT4 may be a potential tumor gene, but the specific expression of ZMAT4 and related studies on the survival and prognosis of patients have not been found in TC clinical samples.

At the same time, with the development of thyroid carcinoma group, prompt ZMAT4 may be a tumor suppressor gene which produces certain effect to thyroid cancer occurrence and development [11]. The expression level of ZMAT4 messenger ribonucleic acid (mRNA) in papillary carcinoma patients is more obvious, but no study has detailed the reasons [12]. The reduced survival rate and other adverse outcomes of patients with thyroid cancer are associated with high expression of ZMAT4 [13]. ZMAT4 gene is a potential tumor gene. The results of its expression alone or in combination with other markers have important reference significance for the diagnosis of hematological malignancies, so the expression level of ZMAT4 has a high auxiliary reference value in the generation, deterioration, and subsequent staging diagnosis of TC.

## 3. Observation Indicators and Statistical Processing

The clinical data related to TC are retrieved and downloaded from TCGA, and the patients corresponding to the data are followed up until December 2021. A total of 389 TC patients related to ZMAT4 gene and its corresponding clinical data are selected and included in the TC group, including 176 males and 213 females. The age ranges from 18 to 68 years, with an average of (48.53 ± 14.36) years. In addition, 76 matched normal tissues are selected and included in the control group, including 28 males and 48 females, aged from 27 to 67 years, with an average of (46.43 ± 12.39) years. All patients enrolled in the study signed informed consent forms.

Inclusion criteria contain the following:

1. Meet the clinical diagnostic criteria for TC.
2. Complete clinical data and general information.
3. Signing informed consent.
4. Have high research compliance and can cooperate with research.

Exclusion criteria contain the following:

1. Combined with other types of tumor.
2. People with mental diseases.
3. Lack of clinical data prevents research.

RT-PCR is used to detect ZMAT4 gene in T cells of TC patients. RNA extraction includes the following steps:

1. Separate radioligand therapy (RLT) solution according to the number of samples: take RLT solution out of the kit and divide it into 1.5 mL centrifuge tubes, 500 *μ*L each.
2. Add thyroid cancer tissue into RLT liquid tube, mix thoroughly, add 5 *μ*L *β*-mercaptoethanol to each tube, then add 600 *μ*L 70% ethanol in turn, and mix thoroughly.
3. Take out the 2 mL collection tube with filter column from the kit and open the package and mark it. Add 600 *μ*L of the mixture in step (2) to the filter column, centrifuge at 12000 rpm for 15 s, and discard the centrifugal liquid in the collection tube.
4. Put the filter column back on the collection tube, and all the mixture remaining in step (2) is sucked into the filter column and centrifuged at 12000 rpm for 15 s, and the centrifugal liquid is discarded.
5. 700 *μ*L wash buffer RW1 is added to the filter column and centrifuged at 12000 rpm for 15 s.
6. Take a clean 2 mL collection tube from Qiagen RNeasy Mini Kit, move the centrifuged filter column to the new collection tube, add 500 *μ*L wash buffer RPE solution to the filter column, 12000 rpm, and centrifuge for 15 s.
7. Discard the centrifugal liquid in the collection tube, then add 500 *μ*L wash buffer RPE solution to the filter column, and centrifuge for 2 min at 13000–14000 rpm.
8. Move the filter column to a clean 1.5 mL Eppendorf tube, add 30∼50 *μ*L rnase-free water to the filter column and stand for 1∼3 min at room temperature.
9. Centrifuged at 12000 rpm for 1 min, the centrifuge solution is collected as the extracted ZMAT4 RNA, which is immediately tested or stored below −20°C.

Reaction system configuration includes the following steps:

1. Negative control: sterile water; positive control: known ZMAT4 RNA.
2. The reaction solution is mixed and divided into 0.2 mL polymerase chain reaction (PCR) tubes, 20 *μ*L for each tube, and labeled, respectively.
3. Add RNA template.
4. Add the assembled PCR tubules into the template. First, add negative control with 5 *μ*L sterile water, then add sample RNA with 5 *μ*L per tube, and finally add positive control RNA with 5 *μ*L per tube.

RT-PCR reaction and product detection include the following steps:

1. Mix the reaction tube with the template and put it into the PCR instrument for RT-PCR amplification after a short centrifugation.
2. Preparation of 2.0% agarose gel: 2.0 g agarose is weighed and poured into a heat-resistant glass jar, and then 100 mL electrophoresis solution (1 × TBE) is added, mixed gently, and heated to melt agarose completely. After agarose cools, add the nucleic acid dye and mix well. When the glue temperature drops to about 50 °C, pour it into the glue making board and insert it into an electrophoresis comb. Pull out the comb after the glue is completely solidified.
3. Put the prepared gel into the electrophoresis tank and pour into the electrophoresis solution.
4. Take 10 *μ*L of PCR products, add 2 *μ*L of sample loading buffer, mix well and add electrophoresis gel, and then add sample PCR products.

The technical route of this study is shown in Figure 1.

The observation indicators are as follows:

1. The difference of ZMAT4 gene expression between normal thyroid tissue and TC tissue is compared.
2. The clinical case parameters of TC patients in the low expression group and the high expression group are compared.
3. The survival curve is drawn to observe the prognosis and survival of TC patients with different ZMAT4 gene expression.
4. Survival curve is drawn to observe the relationship between ZMAT4 expression level and prognosis and survival of TC patients with different clinicopathological characteristics. The predictive value of ZMAT4 gene for the prognosis of TC patients is evaluated by the receiver operating characteristic (ROC) curve.

All data in the study are put into SPSS 25.0 statistical software for data analysis:

1. Measurement data: normality test is performed on the data first. If the data follow normal distribution and homogeneity of variance, they are represented by ($\overset{–}{x}$ *±* *s*). Paired sample *T* test is used to test within the group, and variance comparison is used between groups.
2. Count data: descriptive statistical analysis is conducted by percentage, and *x2* test is performed.
3. Survival analysis: Kaplan–Meier survival curve is drawn for the prognosis and survival of patients in the two groups. *P* < 0.05 indicates significant difference.

## 4. The Prognosis and Survival of TC Patients and ROC Evaluation

### 4.1. Comparison of ZMTA4 Gene Expression Differences

Table 1 shows the comparison of ZMTA4 expression levels. It is clearly evident from Table 1 that the expression level of ZMAT4 gene in TC tissues is lower than that in normal tissues (*P* < 0.05).

### 4.2. Relationship between Different ZMAT4 Gene Expression Levels and Clinical Case Characteristics

Table 2 shows the relationship between ZMAT4 gene expression levels and clinical case characteristics. It is clearly evident from Table 2 that ZMTA4 expression level is related to tumor node metastasis (TNM) stage, histological type, and N stage (all *P* < 0.05).

### 4.3. The Prognosis and Survival of TC Patients with Different ZMAT4 Gene Expression

Figure 2 shows the relationship between ZMAT4 gene expression levels and clinical case characteristics. It is clearly evident from Figure 2 that survival rate of TC patients with low ZMAT4 expression is higher than that of TC patients with high ZMAT4 expression (log-rank = 15.779, *P* < 0.001).

### 4.4. The Relationship between ZMAT4 Expression Level and Prognosis

Figure 3 shows the survival rate of TNM stage I-II patients with different ZMAT4 expression levels. It is clearly evident from Figure 3 that the survival rate of patients with high expression of ZMAT4 is significantly lower than that of patients with low expression of ZMAT4 in TNM stage I-II.

Figure 4 shows the survival rate of TNM stage III-IV patients with different ZMAT4 expression levels. It is clearly evident from Figure 4 that the survival rate of patients with high expression of ZMAT4 is significantly lower than that of patients with low expression of ZMAT4 in TNM stage III-IV.

Figure 5 shows the prognosis and survival of patients with different ZMAT4 expression levels in papillary carcinoma. It is clearly evident from Figure 5 that the survival rate of patients with high expression of ZMAT4 is significantly lower than that of patients with low expression of ZMAT4 in papillary carcinoma.

Figure 6 shows the prognosis and survival of patients with different ZMAT4 expression levels in N0 stage. It is clearly evident from Figure 6 that the survival rate of patients with high expression of ZMAT4 is significantly lower than that of patients with low expression of ZMAT4 in N0 stage.

### 4.5. ROC Evaluation of the Prognostic Value of ZMAT4 Gene

Table 3 shows the diagnostic efficacy. It is clearly evident from Table 3 that ZMAT4 gene has a sensitivity of 82.10% and specificity of 88.30%. The diagnostic efficacy is shown in Table 3.

Figure 7 shows the ROC evaluation of the prognostic value of ZMAT4 gene for TC patients. It is clearly evident from Figure 7 that ZMAT4 gene has a good predictive effect on the prognosis of TC patients.

Through the above experimental results, it can be observed that the expression of ZMAT4 mRNA in thyroid cancer tissues is related to histological type, and the data show that the expression level of ZMAT4 mRNA in papillary carcinoma patients is more obvious, but no study has detailed the reasons. In addition, the results of this study also show that the number of high expression of ZMAT4 mRNA in patients with stage I+II thyroid cancer is significantly higher than that in patients with stage III+IV thyroid cancer.

## 5. Conclusion

In this work, the expression level of ZMAT4 in thyroid cancer tissues was lower than that in normal thyroid tissues. The expression results of ZMAT4 in TC tissues analyzed based on bioinformatics show that its low expression is significantly related to the occurrence and development of TC, and its expression level in TC patients could also be used as a reference index to evaluate the development and prognosis of the disease, with certain clinical application value. Although certain research results have been obtained in this study, there are relatively few clinical studies on the mechanism of ZMAT4 in the development of TC, so the results of this study need to be further studied and demonstrated by other scholars.

## Figures and Tables

**Figure 1:** Technology roadmap.

**Figure 2:** Survival curve.

**Figure 3:** The survival rate of TNM stage I-II patients with different ZMAT4 expression levels.

**Figure 4:** The survival rate of TNM stage III-IV patients with different ZMAT4 expression levels.

**Figure 5:** The prognosis and survival of patients with different ZMAT4 expression levels in papillary carcinoma.

**Figure 6:** The prognosis and survival of patients with different ZMAT4 expression levels in N0 stage.

**Figure 7:** ROC evaluation of the prognostic value of ZMAT4 gene for TC patients.

**Table 1:** Comparison of ZMTA4 expression levels.

Group	Number	ZMTA4
TC group	389	0.27 ± 0.16
Control group	76	16.43 ± 2.32
*t*	–	17.231
*P*	–	<0.0001

**Table 2:** Relationship between ZMAT4 gene expression levels and clinical case characteristics.

	Number (*n* = 389)	High expression group		Low expression group	*x2*	*P*
Gender					0.092	0.762
Male	176	87 (49.43%)	88 (50.57%)		–	–
Female	213	102 (47.89%)	111 (52.11%)		–	–
Age (years)					1.032	0.310
≥40	113	65 (57.52%)	48 (42.48%)		–	–
<40	276	174 (63.04%)	102 (36.96%)		–	–
TNM stage	–	–	–		6.392	0.004
I	134	30 (22.39%)	104 (77.61%)		–	–
II	104	29 (27.88%)	75 (72.12%)		–	–
III	76	17 (22.37%)	59 (77.63%)		–	–
IV	75	20 (26.67%)	55 (73.33%)		–	–
Histological type	–	–	–		8.242	<0.001
Papillary carcinoma	214	45 (21.03%)	169 (78.97%)		–	–
Follicular carcinoma	125	49 (39.20%)	76 (60.80%)		–	–
Tall columnar cell carcinoma	38	6 (17.14%)	32 (84.21%)		–	–
Other	12	2 (16.67%)	10 (83.33%)		–	–
N staging	–	–	–		8.222	0.004
N0	238	81 (34.03%)	157 (65.97%)		–	–
N1	147	30 (20.41%)	117 (79.59%)		–	–
M staging	–	–	–		0.252	0.616
M0	265	18 (6.79%)	247 (93.21%)		–	–
M1	9	1 (11.11%)	8 (88.89%)		–	–
Tumor diameter(cm)	–	–	–		0.463	0.496
≥4	92	16 (17.39%)	76 (82.61%)		–	–
<4	297	43 (14.48%)	254 (85.52%)		–	–
The degree of cure	–	–	–		5.294	0.163
R0	286	218 (76.22%)	68 (23.78%)		–	–
R1, R2	68	46 (67.65%)	22 (32.35%)		–	–
Rx	35	27 (77.14%)	8 (22.86%)		–	–

**Table 3:** The diagnostic efficacy.

	95% CI	Sensitivity (%)	Specificity (%)	AUC	Cutoff value
ZMAT4	0.770–0.923	82.10	88.30	0.847	0.653

## Data Availability

The simulation experiment data used to support the findings of this study are available from the corresponding author upon request.
